# Direct cardiovascular effects of glucagon like peptide-1

**DOI:** 10.1186/1758-5996-5-47

**Published:** 2013-08-29

**Authors:** Asfandyar Sheikh

**Affiliations:** 1 Dow Medical College, Dow University of Health Sciences, Baba-e-Urdu Road, Karachi, Pakistan

## Abstract

Current gold standard therapeutic strategies for T2DM target insulin resistance or β cell dysfunction as their core mechanisms of action. However, the use of traditional anti-diabetic drugs, in most cases, does not significantly reduce macrovascular morbidity and mortality. Among emerging anti-diabetic candidates, glucagon like peptide-1 (GLP-1) based therapies carry special cardiovascular implications, exerting both direct as well as indirect effects. The direct cardiovascular effects of GLP-1 and its analogs remain the focus of this review.

## Article

Cardiovascular disorders (CVDs) are the leading cause of adult mortality and morbidity worldwide, accounting for 17 million deaths (30% of all deaths) in 2008 [1]. CVDs pose a significant economic burden on the healthcare systems of both developing and developed countries. According to an estimate by the American Heart Association (AHA), the annual US medical costs for cardiovascular diseases are likely to increase to over USD 800 billion in 2030, which is nearly triple the amount spent in 2010 (USD 272 billion) [2]. Risk factors of CVDs, which are grouped into modifiable and non-modifiable, include hypertension, smoking, hyperlipidemia, being overweight and having a sedentary lifestyle. Most of these risk factors overlap with those of type 2 diabetes mellitus (T2DM) and past studies have demonstrated such a strong relationship between these two entities that AHA has declared “diabetes *is* a cardiovascular disease” [3].

Recent advancements in healthcare have witnessed an improvement in the prognosis of T2DM patients due to earlier detection and improvements in diabetes care [4]. However, the rationale of intensive anti-diabetic therapy has been challenged in multiple studies. The ACCORD study was conducted on patients with T2DM having HbA1c concentrations >7 · 5% and established cardiovascular disease or ≥2 cardiovascular risk factors in order to determine whether a more intensive therapeutic strategy was associated with a reduction in the rate of cardiovascular events [5]. The study, which ended prematurely due to a higher mortality rate in the intensive treatment group, failed to report significant reduction in major cardiovascular events, giving a notion that intensive therapy was associated with significant harm in high risk patients [6].

Current gold standard therapeutic strategies for T2DM target insulin resistance or β cell dysfunction as their core mechanisms of action. For instance, biguanides and thiazolidinediones, also called “sensitizers”, act by reducing hepatic glucose output and promoting uptake of glucose by the periphery. Similarly, another class of drugs, called “secretagogues”, acts by triggering insulin release from the pancreatic β cells. However, the use of traditional anti-diabetic drugs, in most cases, does not significantly reduce macrovascular morbidity and mortality. This notion has led researchers into searching for alternatives that provide substantial benefits without the added side effects. This idea is especially significant because of the fact that T2DM and cardiovascular diseases are almost invariably related. Among emerging anti-diabetic candidates, glucagon like peptide-1 (GLP-1) based therapies carry special cardiovascular implications (Figure 1).

**Figure 1:** **Cardiometabolic actions of GLP-1 and GLP-1 agonists **[7]**.**

### The incretin effect

It is a well-known fact that oral administration of glucose is a more potent stimulus for insulin secretion than parenteral infusion [8]. This notion implies the presence of an accessory secretory stimulus from the gastrointestinal tract, unrelated to blood glucose levels. The term “incretin effect” refers to a concept which postulates that a family of endocrine factors is responsible for inducing an insulin response before a rise in blood glucose levels [9]. However, the term is somewhat vague, given the fact that incretins have been increasingly reported to have certain non-glucose-lowering functions such as the expansion and preservation of pancreatic β cell mass, bone metabolism, neuroprotection and cardioprotection [10,11].

The main hormones in the group include glucose-dependent insulinotropic polypeptide (GIP) and glucagon-like peptide-1 (GLP-1). GIP is a 42 amino-acid peptide hormone released from the K cells of the proximal intestine. Although the main action of GIP is to provide a stimulus for the release of insulin after an oral glucose challenge, the hormone has also been reported to promote lipid uptake in adipocytes [12]. GIP has also been found to exert influence over other tissues such as bone, although its extraglycemic profile is quite limited and largely pre-clinical in nature compared to its much celebrated partner GLP-1 [13].

GLP-1 is a derivative of the transcription product of proglucagon gene and is synthesized mainly by the L cells of ileal mucosa. The full length N-terminal extended forms of GLP-1 (1–37 and 1–36) are biologically inert. However, removal of the first 6 amino acids yields shorter compounds (7–37 and 7–36) that have enhanced biological activity [14]. Further cleavage of the first two N-terminal amino acids results in the formation of GLP-(9–36) which is the major circulating form [15]. Like GIP, GLP-1 is released in response to ingestion of nutrients and acts on pancreatic β cells to stimulate insulin secretion. Both have short half-lives because of rapid enzymatic inactivation mainly by dipeptidyl peptidase-4 (DPP-4). However, unlike GIP, GLP-1 has not been found to have a direct role in fat deposition in adipose tissues [16]. Furthermore, while GIP augments postprandial glucagon response, GLP-1 extenuates it [17-19]. Similarly, GIP promotes bone formation while GLP-1 inhibits it [20]. Both GIP receptor (GIPR) and GLP-1 receptor (GLP1R) belong to the G-protein coupled receptor family that function by activating adenylate cyclase causing increased levels of intracellular cyclic adenosine monophosphate (cAMP) and activation of protein kinase A (PKA) [21]. Both have been found to be associated with improved cognitive function due to their expression in brain tissue [22-24]. However, unlike GIPR, GLP-1R are present in several other tissues such as peripheral nervous system, lung and heart (Figure 2) [19].

**Figure 2:** **Mechanism of action of GLP-1 **[25]**.**

GLP-1 based anti-diabetic therapies may be divided into two main groups: GLP-1 agonists and DPP-4 inhibitors (Figure 3). Exenatide and liraglutide, which belong to the first category, have already been approved by the FDA for the treatment of T2DM. These drugs are homologous (53% and 97% respectively) to natural GLP-1, with the added benefit of resistance to degradation by DPP-4 which enhances their half-life. Sitagliptin, vildagliptin, saxagliptin and linagliptin (DPP-4 inhibitors) have also been FDA approved, while others are undergoing trials [26]. The prospects for these drugs are quite exciting, especially for those with superimposed CVDs, given the fact that these drugs provide an added advantage of cardioprotection via different yet intricately related mechanisms.

**Figure 3:** **Cardiovascular effects of DPP-4 inhibitors **[27]**.**

### Direct cardiovascular effects of GLP-1

Previous researches have demonstrated the presence of high-affinity receptors for GLP-1 in both human and animal models of hearts and vascular tissues, although the receptors were not localized until later by Ban et al. to cardiomyocytes, endothelium, and vascular smooth muscle cells [28-31]. The presence of these receptors suggests the possibility of prospective drug targets for heart failure and other CVDs both in the presence or absence of pre-existing T2DM.

### Effects on myocardium

#### Electrophysiologic effects

GLP-1 infusions in murine models have been reported to cause a dose-dependent inotropic and chronotropic effect. However, the existence of direct effects on cardiovascular system remains controversial due to conflicting results for in vivo and in vitro studies. For example, Barragan et al. and Yamamoto et al. demonstrated sympathomimetic mechanisms to be responsible for inotropic and chronotropic effects in murine models in vivo, and others such as Ahren et al. demonstrated similar effects that were not suppressed by reserpine, propranolol, or phentolamine, thereby suggesting a direct mode of action [32-34]. These findings was further supported by the study of Gros et al. who demonstrated a diminished basal heart rate and diastolic dysfunction after insulin administration in GLP-1R knockout mice [35]. However, experiments conducted in other settings have yielded contradictory results. For example, Deacon et al. failed to demonstrate similar effects in pig models while Vila Petroff et al. reported negative inotropic effects in rat myocyte cultures [36,37]. Similarly, cardiovascular benefits independent of GLP-1R activation have also been demonstrated [38].

Findings from human trials have demonstrated only a modest effect of GLP-1 analog administration on heart rate. In a placebo-controlled trial conducted on subjects with T2DM already receiving anti-diabetic therapy, exenatide administered subcutaneously demonstrated no clinically significant effects on heart rate [39]. Exenatide and liraglutide have been found to have no significant effect on QT interval in trials using moxifloxacin as a positive control [40]. Similar effects have been noted with DPP-4 inhibitors such as sitagliptin and vildagliptin, whereby supratherapeutic doses have succeeded in producing only a minor increase in the QT intervals [41,42].

The effects of GLP-1 infusion have also been studied on animal models of arrhythmias. Dokken et al. observed an amelioration of coronary flow reserve on administration of GLP-1 in pigs with a few minutes of untreated ventricular fibrillation followed by resuscitation [43]. However, no significant improvement was found in myocardial function [43]. Similar findings were reported by who attributed the improvement in coronary function to reduced markers for reactive oxygen species [44]. Human studies on the potential uses are scarce. A study conducted on patients scheduled to undergo coronary artery bypass graft demonstrated reduced occurrence of arrhythmias in those infused with GLP-1 compared with controls [45]. A patent has been registered for treatment of arrhythmias with GLP-1 agonists [46].

### Cardioprotective functions during ischemia/reperfusion

Various theories have been put forward to explain the protective effects of GLP-1 on myocardium. The most upheld revolves around cardiac metabolism [47]. Under normal physiological conditions, cardiomyocytes utilize fatty acids as a fuel for energy [48]. During acute ischemia, they switch to carbohydrate metabolism, which eventually leads to insulin resistance [48]. GLP-1 analogs, such as liraglutide, have been shown to ameliorate insulin resistance and inflammation in previous studies [49]. This attenuation of insulin resistance, therefore, plays a favorable role in cardioprotection [50]. Another proposed mechanism that involves improved glucose uptake is related to the increase in glucose transport proteins (GLUT-2 and GLUT-4) by GLP-1 [51]. In patients with T2DM, GLUT-4 expression is markedly reduced, and GLP-1 mediated up-regulation of GLUTs, especially in cardiomyocytes, helps preserve their integrity [52]. GLP-1 has also been demonstrated to decrease lactate and pyruvate concentrations, thereby providing another mechanism for cardioprotection via improvement in metabolism [53].

Anti-apoptotic mechanisms have also been proposed. The first mechanism involves activation of cAMP and PI-3 K pathways via GLP-1R [54]. Bose et al. demonstrated a reduction in infarct size on administration of GLP-1 both in vitro and in vivo. This effect was abrogated in the hearts in vitro by GLP-1 receptor antagonist, cAMP inhibitor and PI-3 K inhibitor [55]. Other pathways and mediators have also been demonstrated to play a role. For example, Bose et al. demonstrated inhibition of GLP-1 mediated cardioprotection after administration of rapamycin, suggesting a role of mTOR/p70s6 kinase pathway. In an experimental study conducted by Noyan-Ashraf and colleagues, Liraglutide upregulated the independent expression of cardioprotective genes, including Akt, PPARβ-δ, Nrf-2, and HO-1, while suppressing the expression of GSK3β and activation of caspase-3 in murine hearts [56]. This effect was also found to be superior to metformin’s in diabetic mice hearts [56]. Exenatide, another GLP-1 analog, has also been shown to provide cardioprotection via similar mechanisms [57]. Timmers et al. reported reduction in myocardial infarct size and prevention of deteriorated cardiac function on exanatide treatment in porcine model of ischemia/reperfusion [58]. This was associated with an increase in phosphorylated Akt and Bcl-2 expression as well as superoxide dismutase and catalase activity, and a decrease in active caspase 3 expression. Serum insulin levels were also increased without a corresponding change in glucose levels. The cardioprotective function of exendin-4 during hyperglycemic states was further elaborated in a recent study conducted by Younce, whereby exendin-4 was found to improve cardiac function by inhibiting thapsigargin-mediated decrease in SERCA2a mRNA and via active phosphorylation of phospholamban [59]. Sitagliptin and vildagliptin have also been shown to reduce infarct size in various animal studies [60-62]. Anti-inflammatory mechanisms via attenuation of neutrophil activation were demonstrated by Dokken et al. in a rodent ischemia-reperfusion model, who reported a reduced expression of CD11b in rats receiving GLP-1 therapy [63].

Human studies have also provided evidence for cardioprotective functions of GLP-1 analogs and DPP-4 inhibitors in both diabetics and non-diabetics, although larger, randomized trials are still required. In the EXAMI study, Bernink et al. demonstrated that although high dose exenatide treatment did not exercise a significant effect on left ventricular function or area at risk, a trend was observed towards a smaller infarct size as percentage of the area at risk in patients with first acute myocardial infarction who were to be treated with primary percutaneous coronary intervention [64]. Lonborg and colleagues demonstrated a reduction in infarct size and increased myocardial salvage on exenatide administration in a randomized, placebo-controlled trial in human subjects with ST elevation myocardial infarction undergoing primary percutaneous coronary intervention [65]. Improvements in regional and global left ventricular function were observed by Nikolaidis et al. in human subjects with acute myocardial infarction infused with native recombinant GLP-1 for 72 hours following angioplasty [66]. These effects were independent of location of infarct or diabetic status of the patients [66]. Similar effects were demonstrated by investigators, both before and after revascularization procedures [67,68]. In a retrospective analysis of the IMS LifeLink™ database conducted by Best et al., patients on exenatide were less likely to have a major cardiovascular event, and had reduced risk of hospitalization compared with those receiving other anti-diabetics [69].

DPP-4 inhibitors have also shown encouraging results in human studies. In a placebo-controlled trial conducted on patients having pre-existing coronary artery disease with preserved left ventricular function, increase in GLP-1 levels caused by DPP-4 inhibition resulted in improvement of global and regional left ventricular function and amelioration of post-ischemic stunning [70]. New horizons are being explored in this regard, with a recent study providing promising results in the combination trial (SITAGRAMI-Trial) of sitagliptin and G-CSF based stem cell mobilization [71].

### Cardioprotective functions in heart failure

Both preclinical and clinical studies have demonstrated beneficial effects of GLP-1 on the failing heart. Most of these studies identify attenuation of insulin resistance as the primary mechanism of action [72]. In a study published in 2004, Nikolaidis et al. demonstrated improvement of cardiac output, systolic/diastolic function and other hemodynamic parameters after infusion of recombinant GLP-1 in canine models of pacing-induced dilated cardiomyopathy [50]. These results were further supported by another study from the same lab, whereby GLP-1 was shown to stimulate myocardial glucose uptake via mechanisms that were p38α MAP kinase and NO dependent, but independent of adenylyl cyclase or Akt [73]. These results have been successfully replicated in studies using other animal models. Vyas et al. reported improved glucose tolerance, cardiac contractility, and survival after infusion of exenatide in murine model of dilated cardiomyopathy [52]. Although the expression of myocardial GLUT4 was upregulated, no significant differences were found in the total myocardial GLUT1 levels between groups [52]. Another important finding of this study was that exenatide was also found to abolish the harmful effects of ritonavir (GLUT4 antagonist) on survival [52]. Poornima et al. demonstrated greater survival, preserved LV function, decreased myocyte apoptosis and reduced caspase-3 activation on chronic GLP-1 infusion in spontaneously hypertensive, heart failure prone rats [74]. Additionally, increased plasma insulin, decreased triglycerides, and improved myocardial glucose uptake were observed in the GLP-1 treated group [74]. Similar results were reported by Liu and colleagues [75].

DPP-4 inhibition has also yielded positive results. For example, Shigeta et al. observed reversal of diastolic ventricular dysfunction in a rat model due DPP4 inhibition, via local actions on angiogenesis and inotropic effects [76]. Similar results were reported by Gomez et al. who observed preservation of glomerular filtration rate, increase in stroke volume, and enhancement of the inotropic effect of exogenous brain natriuretic peptide due to DPP-4 inhibition [77].

Earlier studies have hinted towards improved myocardial function with reasonable tolerability in heart failure patients infused with GLP-1 [78]. For example, Sokos et al. reported improved left ventricular ejection fraction, myocardial ventilation oxygen consumption, 6-minute walk distance and quality of life in both diabetic and non-diabetic, class II/IV heart failure patients infused with GLP-1 [79]. However, Halbirk et al. reported only minor cardiovascular effects despite increased insulin levels and reduced plasma glucose concentration, in patients without diabetes but with compensated heart failure [80]. Similarly, in another study conducted by Nathanson et al., infusion of exenatide in male type 2 diabetic patients with chronic heart failure exhibited positive chronotropism and favorable effects on the cardiac index and hemodynamics; however, the definitive effects of exenatide in such patients were still inconclusive [81]. This notion implies that, although favorable results have been reported for clinical studies, the paucity of existing data warrants the need for further ventures in order to further elucidate the favorable effects of GLP-1 in heart failure patients [82].

### Effects on vasculature

#### Vasoprotective actions against endothelial dysfunction and atherosclerosis

Endothelial dysfunction, characterized by impaired vasomotility and an increase in pro-coagulant and pro-inflammatory mediators, is a key feature of T2DM [83]. The robust relationship between these two entities has been largely attributed to oxidative stress caused by hyperglycemia, although a few studies have failed to demonstrate a significant reduction in cardiovascular risk as a result of intense glycemic control [84-86]. A strong association also exists with obesity and insulin resistance [87].

Atherosclerosis is the hardening of arterial wall due to progressive accumulation of fatty substances. It is caused by the interplay between endothelial cells, vascular smooth muscle and macrophages. Since reduced anti-coagulant properties and increased pro-inflammatory mediators and reactive oxygen species play important roles in the development of both endothelial dysfunction and atherosclerosis, the association between the two is almost ubiquitous [88].

Newly published reports are improving our understanding of the role of GLP-1 and its analogs in the improvement of endothelial function. For example, in a study conducted by Nathanson et al. on rat conduit arteries ex vivo, exenatide was not found to significantly ameliorate triglyceride-induced endothelial dysfunction nor did it exert a potent vasorelaxant effect [89]. However, contrasting results were found by Goyal et al. who reported improvement in acetylcholine-induced endothelium relaxation on administration of exendin-4 in rat model of T2DM [90]. This effect was abolished by an inhibitor of NOS, suggesting the activation of eNOS by exendin-4 [90]. These results were again contradicted by Murthy et al. who found no significant changes in eNOS and NFkappaB-p65 expression in exenatide treated non-diabetic rats [91]. However, a more recent study conducted by Ding et al. on human umbilical vein endothelial cells (HUVEC) has demonstrated upregulation of eNOS expression via GLP-1R dependent pathways [92].

GLP-1 and its analogs have also been found to inhibit cellular migration and other essential facets of inflammation, thus mitigating atherosclerosis. Nagashima et al. observed inhibition of macrophage foam cell formation by both GLP-1 and GIP, followed by cAMP activation [93]. These effects were found to be associated with downregulation of CD36 and ACAT-1 [93]. Similarly, exendin-4 was demonstrated to inhibit inflammatory response in macrophages by Arakawa et al. [94]. Shiraishi and colleagues demonstrated upregulation of alternatively activated macrophage-related molecules, such as IL-10, CD163, and CD204 in human monocyte-derived macrophage by GLP-1 [95]. GLP-1 also activated STAT3 in a GLP-1R dependent manner [95]. GLP-1 also exerts influence on inflammatory mediators. For example, Liu et al. demonstrated inhibition of TNF-α mediated PAI-1 induction, ICAM-1 and VCAM-1 expression by liraglutide in HUVEC [96]. However, a recent study by Panjwani et al. has provided contradictory results. Taspoglutide (a long acting GLP-1 agonist) was not found to have significant anti-atheromatous effects, although it did reduce hepatic triglyceride levels, suggesting an indirect mode of action [97]. DPP-4 inhibitors have also been shown to have anti-inflammatory actions. Recent studies have demonstrated direct suppression of aortic atherosclerosis by both PKF275-055 and sitagliptin [98-100].

GLP-1 has been shown to confer protective effects on the endothelium and to maintain its integrity. For example, Oeseberg showed that dipeptidyl-peptidase 4 (DPP-4) inhibition significantly reduced vascular senescence in a diabetic rat model. This effect was mediated via activation of cAMP response element-binding transcription factor in a cAMP/PKA-dependent manner and induction of oxidative defense genes HO-1 and NQO1 [101]. Similarly, Goto showed that exendin-4 reduced intimal thickening after vascular injury by the suppression of platelet-derived growth factor-induced proliferation in isolated murine, rat and human aortic vascular smooth muscle cells [102]. In vitro studies in HUVECs have further demonstrated these effects. In a study by Ishibashi et al., GLP-1 was shown to dose-dependently inhibit gene expression for advanced glycation end products receptor (RAGE) in HUVEC via activation of cyclic AMP pathways and decrease reactive oxygen species generation [103]. This effect was directly mediated via the GLP-1R [103]. In another study, liraglutide was shown to prevent the onset of endoplasmic reticulum stress in HUVECs exposed to high glucose via dose dependent induction of mitochondrial fusion marker, OPA1, thereby inhibiting mitochondrial fragmentation and apoptosis [104]. Liu and colleagues showed that GLP-1 suppressed the oxidized low-density-lipoprotein-induced apoptosis of MILE SVEN 1 cells by inactivating the PARP-1/iNOS/NO pathway [105]. This effect was accompanied by a significant decrease in intracellular nitric oxide activity, suppression of lipid peroxidation and restoration of the activities of endogenous antioxidants [105]. Ergogdu showed that incubation of human coronary artery endothelial cells (HCAECs) with exendin-4 caused an increase in DNA synthesis and cell proliferation through PKA-PI3K/Akt-eNOS activation pathways via a GLP-1 receptor-dependent mechanism [106]. Another paper by the same group showed that incubation of HCAECs with exendin-4 resulted in a dose-dependent up-regulation of DNA synthesis which was associated with enhanced eNOS and Akt expression [106]. This effect was inhibited by PKA, PI3K, Akt or eNOS inhibitors and abolished by a GLP-1 receptor antagonist. Human studies have also demonstrated beneficial effects. For example, Ceriello et al. reported that during the meal, GLP-1 exerted simultaneous effects on insulin secretion and endothelial protection, in a manner dependent on the level of glycemia [107]. Additional data show that liraglutide reduces several markers of cardiovascular risk, such as body weight, A1C levels, Systolic BP, C-reactive protein, type 2 natriuretic peptide, and PAI-1 [108,109]. Exenatide has also exhibited similar effects, with efficacy comparable to that of metformin [110].

### Regulation of vasomotor functions and arterial blood pressure

GLP-1 has been demonstrated to modulate peripheral arterial blood flow by exerting direct effects or via signals from the CNS. Richter showed that addition of GLP-1 caused increase in 35S-sulfate-labeled macromolecule secretion and relaxation of the pulmonary artery [111]. He concluded that GLP-1 may act as neurotransmitter of the peptidergic nervous system in airways [111]. Similarly, Golpon also showed the role of GLP-1 in the modulation of pulmonary vascular tone [112]. Nystrom and colleagues showed dose-dependent relaxation of femoral artery rings by GLP-1 in a rat organ bath model [113]. This effect was shown to be independent of NO and the endothelium [113]. In contrast, Dong et al. concluded that GLP-1 had a role in expanding microvascular volume via a PKA/NO-dependent pathway in the vascular endothelium [114]. In another study, GLP-1 and exendin-4 treatment was shown to normalize the altered vascular tone in type 2 diabetic rats, with the latter being less effective [115]. In a study published in 2012, Wu hypothesized that the vascular modulatory effect on pancreatic islet microcirculation may in fact be one of the mechanisms for anti-diabetic actions of GLP-1 and exendin-4. She showed that infusion of both GLP-1 and exendin-4 prevented glucose-induced pancreatic blood flow redistribution into the islets, an effect that was not abolished by blocking NO formation [116]. Human studies have also pointed towards amelioration of endothelial dysfunction and modulation of vascular reactivity [117]. In the study conducted by Nystrom, GLP-1 was found to be associated with improvement in endothelial dysfunction without improvements in insulin resistance in T2DM patients with coronary heart disease [118]. Due to the direct and indirect role of GLP-1 on endothelial functions, GLP-1 receptor antagonists may also serve as potential prospects in addressing cardiovascular risks in T2DM patients [119].

GLP-1 has also been shown to regulate peripheral arterial blood flow via signals from the CNS [33,120]. For example, in 2004, Cabou et al. demonstrated that central GLP-1 signaling plays an essential role in the regulation of arterial blood flow, heart rate, and insulin sensitivity [121]. This study was further reinforced by another one in 2011, whereby brain GLP-1 signaling was shown to activate hypothalamic glucose-dependent PKC-δ to regulate femoral artery blood flow and insulin sensitivity [122]. Similarly, Isbil-Buyukcoskun and colleagues showed that intracerebroventricularly injected GLP-1 had a role in increasing blood pressure and heart rate [123]. The former was mediated by stimulation of central nicotinic and partially muscarinic receptors and vasopressinergic system, while the latter was mediated by stimulation of central nicotinic receptors [123].

GLP-1 and its analogs also have potent effects on blood pressure, and may therefore play a role in ameliorating hypertension. Previously published data has demonstrated the GLP-1 analogs to have a direct natriuretic effect and a direct mode of action on endothelial vasodilatation [124,125]. The mechanisms for GLP-1 mediated diuresis and natriuresis were explained by Crajoinas et al., who reported that these effects were mediated by changes in renal hemodynamics and by downregulation of NHE3 activity in the renal proximal tubule [126]. Recombinant GLP-1 was shown by Yu et al. to have an antihypertensive effect in Dahl Sensitive rats fed with a high salt diet, in addition to cardioprotective and renoprotective effects [127]. The antihypertensive effect is due to its diuretic and natriuretic actions, rather than amelioration of insulin resistance [127]. Exendin-4 also has antihypertensive effects in salt-sensitive mice models. Hirata and colleagues demonstrated that exendin-4 attenuated high-salt load induced hypertension, prevented angiotensin II induced hypertension and inhibited angiotensin II-induced phosphorylation of ERK1/2 [128]. Exenatide has also been shown to have an antihypertensive effect in glucocorticoid-induced model of the metabolic syndrome [129]. This effect occurred independently of changes in body weight [129]. DPP-4 inhibitors have also been demonstrated to have an antihypertensive effect. For example, Sitagliptin was shown to increase GLP-1 and GLP-1 receptor expression in spontaneously hypertensive rat renal arteries by Liu [130]. This upregulation was associated with improvement of endothelial function via restoration of NO bioavailability [130]. This effect was further shown to be partially due to inhibition of NHE3 activity in renal proximal tubule [131].

GLP-1 and its analogs have also been demonstrated to have antihypertensive effects in human studies. For example, exenatide intake was associated with weight loss and reduction in levels of HbA1c, systolic blood pressure, triglycerides, and high-sensitivity CRP in obese patients with type 2 diabetes on insulin [132]. The effect on systolic blood pressure was further confirmed by a pooled analysis of 2171 patients [133]. Liraglutide, long-acting GLP-1 agonist, has also been shown to induce significant weight loss and reduce SBP in a group of Asian patients [134]. Antihypertensive effects have also been observed for DPP-4 inhibitors. For example, Yanai et al. reported reduction of body weight, HbA1c levels and blood pressure after 6-month treatment with sitagliptin [135]. The antihypertensive effect of sitagliptin was confirmed by Ogawa, who showed that this effect was independent of BMI and blood glucose reduction [136].

## Conclusion and future directions

Recent studies provide potent evidence for the pleiotropic effects of GLP-1 on the cardiovascular system. This review attempts to highlight the direct cardiovascular effects, without going into details of the indirect actions, which have already been thoroughly reviewed in previous papers. Majority of the present GLP-1 based studies employ GLP-1 analogs such as exenatide as their primary drugs, which raises a question for their cardiovascular safety and contribution to major adverse cardiovascular events (MACE). In an integrated analysis of 3,945 participants, Ratner et al. observed no increase in cardiovascular risk with the use of exenatide BID in patients with type 2 diabetes [137]. Similarly, liraglutide has not been found to be associated with an increase in MACE in FDA’s review as well as in a pooled analysis of phase 2 and 3 clinical trials [138,139]. Its safety has been confirmed by a recent study published in Lancet, whereby liraglutide had an efficacy comparable to that of glimepiride, but was associated with fewer cardiovascular events [140]. DPP-4 inhibitors also have a favorable cardiovascular safety profile [141]. However, the recently concluded SAVOR-TIMI 53 trial conducted on patients with T2DM with either a history of established CVD or multiple CVD risk factors, has failed to demonstrate the superiority of saxagliptin over placebo in reducing a composite end point of cardiovascular death, nonfatal MI or nonfatal ischemic stroke when added to usual care [142,143]. Nevertheless, the relatively low occurrence of MACE implies that the translation of ongoing research to the bedside would provide a safe therapeutic alternative to available anti-diabetics, with additional cardioprotective and vasculoprotective effects.

It is important to note that the dividing line between direct and indirect effects is tenuous and somewhat vague. Its fragility is reinforced by the relative scarcity of existing data that provides conclusive evidence for delineating the two. This notion implies the need for additional preclinical and clinical studies that are focused primarily on distinguishing these two entities. These studies will not only provide therapeutic benefits to T2DM patients with superimposed CVDs, but may also unveil new horizons in cardiovascular research. A search at http://www.clinicaltrials.gov (using keywords GLP-1 and cardiovascular) returns 36 open studies, which hints towards an increasing interest in the cardiovascular effects of incretin based therapies.

## Competing interests

The author declares that he has no competing interests.
